The article "The Prognostic Role of m6A-Related Genes in Paediatric Neuroblastoma Patients" was published in 2022. Journal: Comput Math Methods Med.

# The Prognostic Role of m6A-Related Genes in Paediatric Neuroblastoma Patients

**DOI:** 10.1155/2022/8354932

**Published:** 2022-01-10

**Authors:** Chunyang Zhang, Zhaozheng Ding, Hong Luo

**Affiliations:** ^1^Department of Pediatric Surgery, The First People's Hospital of Lianyungang, Lianyungang, Jiangsu, China; ^2^The First Affiliated Hospital of Kangda College of Nanjing Medical University, China

## Abstract

**Methods:**

The gene expression data were extracted from the “Therapeutically Applicable Research to Generate Effective Treatments” (TARGET) database. The differentially expressed genes (DEGs) were identified, and the relationships between DEGs and m6A genes were explored. Then, the correlations among the m6A genes in neuroblastoma were investigated. Finally, the prognostic role of the m6A genes was studied, and the risk model was constructed.

**Results:**

81 NB patients were extracted from the TARGET database. After comparing the gene expression between unfavorable and favorable outcome groups, 73 DEGs were identified, including 54 downregulated genes and 19 upregulated genes. In NB patients, we found that IGF2BP3, METTL14, and METTL16 are prognostic factors for disease-free survival (DFS) while IGF2BP3, METTL14, and METTL16 are prognostic factors for overall survival (OS). Besides, after the risk model construction, the OS between the two risk groups was drawn (log-rank *p* = 1.64*e* − 08, HR = 3.438, 95% CI 2.24-5.278). The 1-, 3-, and 5-year time-dependent receiving operating characteristic (ROC) curves were also illustrated, and the areas under the receiver operating characteristic curves (AUCs) attained 0.75, 0.798, and 0.768, respectively.

**Conclusions:**

IGF2BP3, METTL14, and METTL16 were identified as the significant factors for DFS and OS in NB patients.

## 1. Introduction

Neuroblastoma (NB) is the most common extracranial solid tumor in children, which originated from sympathetic ganglia and bilateral adrenal glands, and has the highest incidence rate and mortality rate in infancy, accounting for 8%-10% of children's tumors [1]. The incidence of NB is age-related. The average age at the time of clinical diagnosis is 17.3 months, and 40% of children are diagnosed before 1 year old [2]. In terms of survival rate, 85% to 90% of low- and moderate-risk children can be cured, while the survival rate of high-risk NB children is less than 50% [3]. High-risk children with NB are still difficult to cure after repeated intensive treatments. More than 50% of the children relapse, and the 5-year survival rate is about 40% to 50%. Therefore, it is very important to develop new treatments for high-risk NB [4, 5].

The vast majority of NB patients are nonfamilial and sporadic. Only about 1% to 2% of individuals have a family history and are related to specific gene mutations. At present, genes closely related to NB have been found to include MYCN, ALK, ATRX, NRA, and PHOX2B [6]. Among them, MYCN and ALK gene abnormalities are the two most common targets for the treatment of NB [7]. MYCN has a key role in the proliferation, differentiation, metastasis, apoptosis, and angiogenesis of NB cells. Therefore, the MYCN gene has become an important target for the treatment of NB and other related tumors. The ALK gene is the driving gene of primary and recurrent NB, and ALK gene mutation is one of the signs of poor prognosis of NB [8]. Therefore, ALK inhibitors will be an important tool for clinical treatment of NB. The research content of epigenetics studies mainly includes histone modification, DNA methylation, chromatin structure reconstruction, and noncoding RNA regulation. Changes in epigenetics can affect the maintenance of stem cell phenotypes and promote the occurrence of tumors through the synergistic effects of DNA methylation, histone methylation or acetylation, and gene silencing [7, 8].

N6-Methyladenosine (m6A) is the most abundant RNA internal modification in eukaryotic cells, and it has received more and more attention in recent years. High-throughput m6A sequencing studies have shown that m6A modifications, including significant enrichment of 3′ UTR near the stop codon, are widespread at the transcriptome level, affecting thousands of mRNAs and noncoding RNAs. New evidence suggests that m6A methylation plays a key role in cancer through various mechanisms. m6A methylated modification played an important role in several major physiological processes such as brain development, spermatogenesis, hematopoietic stem and progenitor cell specification, and control of the circadian clock [9, 10]. Additionally, m6A methylation markers were reported to be related to the occurrence and development of tumors and had the potential to be used for early tumor screening. These prognostic markers that reflect tumor progression at the molecular level may help to better achieve personalized survival prediction [4]. However, evidence remains insufficient, particularly in paediatric malignant tumors. Here, we systematically analyzed the role of m6A-related genes and explored the clinical significance of m6A-related genes in NB patients.

## 2. Materials and Methods

### 2.1. Differential Gene Identification

From the TARGET dataset (https://ocg.cancer.gov/programs/target), the raw count of RNA sequencing data (level 3) of 181 NB tumors and the corresponding clinical information were obtained. Using the limma package of R software (version 4.0.5) to explore the differential expression of mRNA, “adjusted *p* < 0.05 and log2 | fold change | >1 or log2 | fold change | <−1” is defined as the differentially expressed genes (DEGs) [11].

### 2.2. Function Enrichment

In order to further confirm the potential function of the potential target, the data was analyzed through function enrichment. Gene Ontology (GO) is a widely used tool for annotating functional genes, especially biological pathways (BP), molecular functions (MF), and cellular components (CC) [12]. Kyoto Encyclopedia of Genes and Genomes (KEGG) enrichment analysis is practical and can be used to analyze gene function and related advanced genome function information. In order to better understand the carcinogenic effects of target genes, the ClusterProfiler package is employed to analyze the GO function of potential DEGs and enrich the KEGG pathway.

### 2.3. m6A Gene Extraction

We followed the previous articles [13] and obtained the m6A genes.

### 2.4. Survival Analysis

Disease-free survival (DFS) is defined as the time interval from the time of the first diagnosis to the time of disease relapse. Overall survival (OS) is defined as the time interval from the time of the first diagnosis to the time of death or censored. The survival curves were drawn by Kaplan-Meier curves using the log-rank test [14].

## 3. Results

In general, we extracted 181 NB patients from the TARGET database. Among them, after extended standardization, 133 patients with unfavorable outcomes and 41 with favorable outcomes were finally extracted.

After comparing the gene expression between unfavorable and favorable outcome groups, 73 differentially expressed genes (DEGs) were identified, including 54 downregulated genes and 19 upregulated genes. The heat map (Figure 1(a)) and volcano plot (Figure 1(b)) for the DEGs are drawn. Moreover, we explored the KEGG pathways and GO for the downregulated and upregulated DEGs, respectively (Figure 2). In Figure 2(a), the KEGG pathways and GO analysis for the upregulated DEGs demonstrated that the Fanconi anemia pathway is the most enriched pathway and the top three GO are organelle fission, nuclear division, and chromosome segregation, respectively (Figure 2(a)), while in downregulated DEGs, neuroactive ligand-receptor interaction is the most enriched pathway and the top three GO are cell junction assembly, synapse organization, and synapse assembly, respectively (Figure 2(b)).

Then, we further investigated the relationships between DEGs and m6A genes using the PPI network. We found that DEGs and m6A genes had associations by the genes TTK and MLH1 (Figure 3). We supposed that the m6A genes may have prognostic value for NB patients. First, we conducted a genetic correlation analysis for m6A genes in NB patients. The results are shown in Figure 4. Second, we compared the expression differences of m6A genes between unfavorable and favorable outcome NB groups and illustrated that ALKBH5, ZC3H13, METTL14, YTHDC1, HNRNPA2B1, METTL3, NHRNPC, RBMX, RBM15B, YTHDF1, IGF2BP1, RBM15, and IGF2BP3 are all differentially expressed (Figure 5).

As for survival analysis, in all the NB patients, we found thatIGF2BP3 (log-rank *p* = 0.008, HR = 1.76, 95% CI 1.16-2.67), METTL14 (log-rank *p* = 0.005, HR = 1.84, 95% CI 1.21-2.8), and METTL16 (log-rank *p* = 0.01, HR = 0.579, 95% CI 0.381-0.879) are prognostic factors for DFS (Figure 6) while IGF2BP3 (log-rank *p* = 0.033, HR = 1.55, 95% CI 1.03-2.31), METTL14 (log-rank *p* = 0.038, HR = 1.53, 95% CI 1.02-2.3), and METTL16 (log-rank *p* = 0.003, HR = 0.534, 95% CI 0.354-0.806) are prognostic factors for OS (Figure 7).

We used the least absolute shrinkage and selection operator (LASSO) model to select the optimal genes for constructing the risk model, and we found that when lambda.min = 0.0185, we could obtain the optimal model (Figure 8(a)). The risk score is defined as

(1) $$\begin{array}{c} \text{Riskscore}=\left(0.809\right)*\text{METTL}3+\left(0.5311\right)*\text{METTL}14+\left(-1.3683\right)*\text{METTL}16+\left(-0.0483\right)*\text{ZC}3\text{H}13+\left(0.2584\right)*\text{RBM}15+\left(-0.6633\right)*\text{WTAP}+\left(0.6862\right)*\text{KIAA}1429+\left(0.5209\right)*\text{YTHDF}1+\left(-0.5415\right)*\text{YTHDF}2+\left(-0.9856\right)*\text{YTHDF}3+\left(-0.0044\right)*\text{YTHDC}2+\left(0.3623\right)*\text{HNRNPC}+\left(0.0923\right)*\text{IGF}2\text{BP}2+\left(0.1269\right)*\text{IGF}2\text{BP}3+\left(-0.1131\right)*\text{FTO}. \end{array}$$

We then obtained the high-risk and low-risk groups according to the risk score (Figure 8(b)). The overall survival between the two groups was drawn (Figure 8(c), log-rank *p* = 1.64*e* − 08, HR = 3.438, 95% CI 2.24-5.278). The 1-, 3-, and 5-year time-dependent ROC curves were also illustrated, and the AUCs could reach up to 0.75, 0.798, and 0.768, respectively (Figure 8(d)).

## 4. Discussion

The tumor heterogeneity of NB is closely related to its clinical and biological behavior. The treatment effect of different patients is uneven, especially for the treatment of children with high-risk NB, which lacks targeted methods, resulting in a poor overall prognosis. The study of the NB genome and biological characteristics is of great significance for further elucidating the pathogenesis of NB, exploring potential therapeutic targets, and improving the survival rate of patients [1–4, 15], although a variety of treatment methods have been established for NB, such as surgical resection, chemotherapy, radiotherapy, immunotherapy, and autologous hematopoietic stem cell transplantation [2, 5, 7]. And with the development of multimodal treatment strategies, the OS of low- and medium-risk NB has exceeded 90%. However, the 5-year survival rate of patients with high-risk NB is still less than 50%. Therefore, the further stratification of high-risk NB should be strengthened to individualize the multimodal treatment of NB in high-risk groups [1, 15].

m6A regulatory enzymes consist of “writers” (methyltransferases) METTL3, METTL14, RBM15, WTAP, VIRMA, and ZC3H13, “erasers” (demethylases) FTO and ALKBH5, and “readers” YTHDC1, YTHDC2, YTHDF1, YTHDF2, YTHDF3, IGF2BP1, IGF2BP2, IGF2BP3, HNRNPC, HNRNPG/RBMX, FMR1, and EIF3 [16]. Writers are responsible for catalyzing the formation of m6A modifications, erasers are responsible for removing m6A modifications, and readers are involved in the occurrence and development of human diseases by specifically identifying target RNAs modified by m6A. In this study, IGF2BP3, METTL14, and METTL16 are the key molecules that affect the prognosis of NB patients (IGF2BP1/2/3); insulin-like growth factor-2 (IGF2) mRNA binding protein is the latest reported m6A reader family. It can bind to target mRNAs to enhance the stability and translation of mRNA and protect m6A-modified mRNA from degradation. IGF2BPs are a family of highly conserved single-stranded RNA binding proteins, consisting of 6 typical RNA binding domains, including 2 RNA recognition motif (RRM) domains and 4 K homology domains. IGF2BPs play a carcinogenic effect in cancer cells by stabilizing the methylated mRNA of oncogenic targets (such as MYC) [17]. IGF2BP3 binds to the target mRNA in an n6-methyladenosine- (m6A-) dependent manner and promotes mRNA stability and translation by recognizing m6A modification sites. The KH domain binds directly to m6A RNA, especially the KH3-4 two domains that play an important role in stabilizing RNA. IGF2BP3 can affect gene expression, mRNA methylation, mRNA processing, mRNA splicing, cap-independent positive regulation of translation initiation, mRNA destabilization, and primary miRNA processing. IGF2BP3 is a potential oncogene and is significantly upregulated in a variety of human cancer types. It is associated with aggressiveness and poor prognosis and is associated with poor patient survival. IGF2BP3 can be used to identify patients with early diagnosis of RCC renal cell carcinoma. The high expression of IGF2BP3 indicates the metastasis and poor prognosis of renal cell carcinoma RCC. It can be used as an independent prognostic marker of renal cell carcinoma RCC and is an early systemic treatment. IGF2BP3 has been proven to be a predictor of colon cancer progression and poor survival, and its overexpression promotes the proliferation, migration, and invasion of colorectal cancer. It also plays an important role in breast cancer resistance. High expression of IGF2BP3 is associated with low survival rate of patients with gastric cancer (GC). According to literature reports, IGF2BP3 can promote the carcinogenesis of ovarian cancer and pancreatic duct adenocarcinoma. In pancreatic cancer, the DNA methylation level of IGF2BP3 is significantly reduced, and the expression level of IGF2BP3 is increased, which is related to the poor overall survival of patients. In addition, IGF2BP3 promotes the occurrence of lung tumors by weakening the stability of p53. In addition, IGF2BP3 participates in the fetal adult hematopoietic switch by interacting with the RNA-binding protein Lin28b. In B cell progenitor cells, Lin28b and IGF2BP3 promote mRNA stability.

Methyltransferases include METTL3, METTL14, WTAP, KIAA1429, and so on. METTL14 is one of the components of the m6A methyltransferase complex discovered in recent years [18]. METTL14 can participate in the catalysis of m6A by forming a complex heterodimer structure with METTL3, and METTL14 can also form heterodimers with METTL3 to promote the stability of their respective proteins. METTL14 promotes tumorigenesis by upregulating expression of MYC and MYB in acute myelocytic leukaemia (AML) but acts as a tumor suppressor by inactivating AKT in endometrial cancer. High expression of METTL14 was reported to be significantly correlated with low overall survival of patients with NB, and the high-risk group was highly enriched in MYC targets, suggesting that METTL14 exerted its potential functions through MYC-associated pathways.

METTL16, as a newly identified m6A methyltransferase, is currently seldom studied. METTL16 has been proven to be associated with the occurrence and development of a variety of cancers [19]. METTL16 gene deletion indicates poor overall survival and disease-free survival of patients with liver cancer. In addition, METTL16 gene deletion is an independent factor affecting DFS. Breast cancer patients with high METTL16 expression have a lower survival rate, and breast cancer patients with relatively low METTL16 expression have poor recurrence-free survival. Bioinformatics analysis found that METTL16 is expressed in large amounts in colon cancer, but not in rectal cancer. Poor prognosis of colon cancer may be closely related to total m6A levels, including METL3, METL16, and WTAP. In soft tissue sarcoma, patients with increased METL16 expression have a poorer overall survival, and patients with high METL16 expression have more related reflection characteristics. In the studies of four endocrine tumors, the expression level of METTL16 was positively correlated with overall survival. It was observed that METTL16 plays an important role in the development of endocrine system tumors, and METTL16 is a protective gene [20]. Nevertheless, several limitations should be noted. Currently, there are relatively few studies on m6A methylation. Therefore, in order to improve the accuracy of the risk model, additional m6A regulatory factors need to be added. Future biological experiments are necessary. In addition, the genetic characteristics identified as independent prognostic factors in this study are based on the target database, so additional datasets are needed to validate our findings.

In conclusions, we found that in NB patients, IGF2BP3, METTL14, and METTL16 were identified as the significant factors for DFS and OS in NB patients. These findings could provide new insights into the potential targets for NB treatment, especially for high-risk patients.

## Figures and Tables

**Figure 1:** Differential analysis. (a) Hierarchical clustering analysis of genes, which were differentially expressed between NB patients with favorable and unfavorable outcomes. (b) Volcano plots for the DEGs.

**Figure 2:** KEGG pathways and Gene Ontology analysis for DEGs: (a) the KEGG and GO analysis for upregulated DEGs; (b) the KEGG and GO analysis for downregulated DEGs.

**Figure 3:** PPI network for DEGs and m6A-related genes.

**Figure 4:** A heat map of the correlation among m6A-related genes. Green represents a positive correlation, and red represents a negative correlation.

**Figure 5:** A heat map for high-risk and low-risk NB patients using m6A genes.

**Figure 6:** Kaplan-Meier survival curves for DFS: (a) IGF2BP3; (b) METTL14; (c) METTL16.

**Figure 7:** Kaplan-Meier survival curves for OS: (a) IGF2BP3; (b) METTL14; (c) METTL16.

**Figure 8:** Patient risk stratification for NB patients: (a) coefficients of m6A genes are shown by the lambda parameter; (b) prognostic analysis of gene signature in the TARGET cohort; (c) Kaplan-Meier survival curves for survival according to the risk stratification; (d) time-dependent ROC analysis of the m6A genes.

## Data Availability

The datasets generated and analyzed during the present study are available in the TARGET database (https://ocg.cancer.gov/programs/target).
